# Prediction Model of International Trade Risk Based on Stochastic Time-Series Neural Network

**DOI:** 10.1155/2022/3119535

**Published:** 2022-06-16

**Authors:** Lei Xu, Guicai Dong

**Affiliations:** School of International Trade and Economics, Anhui University of Finance and Economics, Bengbu, Anhui 233030, China

## Abstract

With the extreme deterioration of domestic and foreign trade environment, international competition is becoming increasingly fierce. At the same time, many enterprises have loopholes in industrial structure and finance, resulting in many risks in their international trade. Therefore, we must take corresponding measures to effectively manage and avoid risks and realize the healthy and sustainable development of foreign trade enterprises and enterprise economy. This paper designs and proposes a risk prediction model combining ARIMA and BP neural network. The model can get good prediction in different time series and effectively avoid the risk. The model proposed in this paper optimizes the structure of the design model with the support of ARIMA algorithm and BP neural network algorithm and has good accuracy and error control for different time series. The purpose of establishing time series prediction model is to improve the prediction accuracy of the model, and it is also an effective way to enhance the practicability of the prediction model. Applying intersequence analysis method to financial risk prediction can greatly improve efficiency and save cost and has broad application prospects.

## 1. Introduction

With China's accession to the international trade organization, import and export enterprises need to participate in the cruel competitive environment of domestic and international markets at the same time. Therefore, the market competition faced by Chinese enterprises is relatively fierce [1]. In addition, based on the continuous changes in the internal and external environment, the daily operations of import and export enterprises are increasingly affected by uncertain factors. Compared with the previous market environment, the current import and export enterprises have increased risk factors [2]. Therefore, by strengthening the risk prediction of international trade import and export enterprises and taking corresponding prevention and control measures, the efficiency of international trade risk prevention and management can be improved, which can meet the requirements of international development and realize the sound development of import and export enterprises.

Because some superior properties of human brain are unmatched by current machines, in order to improve the ability of artificial machines, people gradually form a new discipline of artificial neural network through the exploration and simulation research on the organizational structure and working mechanism of human brain and with the help of mathematical and physical methods [3]. Time series data refers to the sequence formed by the values of different indicators of an object or phenomenon at different times arranged in chronological order. This way of recording data is the most commonly used in actual production and life [4]. The analysis methods of time series mainly originated from the stochastic process theory and statistics category. By studying the statistical laws followed by data series, we can provide guidance for actual production and life [5]. Time series data itself can also be regarded as a dynamic system. Because it is influenced by many factors and then has complex fluctuation characteristics, it is extremely difficult to make effective and accurate prediction for time series data [6]. Prediction refers to the establishment of a system model based on the study of historical events, so as to predict the events with adverse consequences in the future [7]. With the continuous progress of science and technology, prediction methods have also been greatly developed, and various prediction methods emerge endlessly.

In prediction experiments, due to the different modeling mechanisms and the basic points of consideration, there are usually many different prediction methods that can be used for a prediction problem. It is difficult to select the optimal one under comprehensive consideration. The combined forecasting method formed by orderly organization in a reasonable way will be beneficial to comprehensively utilize the information provided by various single forecasting methods and improve the reliability and accuracy of model forecasting, and its performance is often better than that of a single forecasting method [8]. A method to achieve this goal in direct laser writing is proposed, which is an additional manufacturing method based on photopolymerization, which is usually affected by strong shrinkage induced effect [9]. Point prediction is to use the trained model to obtain the predicted value at the specific time point in the future and give specific guidance to the development of future trend. However, this process will be disturbed by many random factors and unpredictable shocks, resulting in difficulty in obtaining convincing prediction results. Interval prediction obtains a numerical interval that the predicted value at the future time may fall into, and its understanding method is similar to the confidence interval in statistics [10]. Probability density prediction refers to the probability distribution or density function to which the predicted value of the future time can be obtained. Similar to interval prediction, it can also give richer information than point prediction.

Aiming at different types of prediction models, such as linear or nonlinear, single or combined, and deterministic or nondeterministic prediction models, it is necessary to study the rationality of the model effect. At present, fractal analysis based on most time series data is based on single fractal theory [11]. This theory is more suitable for simulating stationary time series, because they have only one scale characteristic and their properties are constant [12]. In order to adapt to the dynamics research of complex systems, it is necessary to analyze more scaling indices and to explore the characteristic parameters of time series data from various aspects. By analyzing the business situation of international trade enterprises, this paper finds out the types of risks that may be faced, analyzes the causes of risks and puts forward corresponding solutions, classifies, evaluates, quantitatively and qualitatively studies the risks in international trade, controls the risks in international trade within the acceptable range of enterprises, and strives to coordinate and adapt to the overall development goals of enterprises, so as to ensure the true connection and intercommunication of internal and external information of enterprises, thus improving the efficiency of business operations and promoting the effect of achieving business goals and reducing the risks caused by enterprise decisions.

At present, the research on various combination prediction models has its own shortcomings and deficiencies. This paper designs and proposes a risk prediction model combining ARIMA and BP neural network. The model can get good prediction in different time series and effectively avoid the risk. The innovation contribution is that the model proposed in this paper optimizes the structure of the design model with the support of ARIMA algorithm and BP neural network algorithm and has good accuracy and error control for different time series. The purpose of establishing time series prediction model is to improve the prediction accuracy of the model, and it is also an effective way to enhance the practicability of the prediction model. However, due to the different characteristics of various prediction methods, the prediction effect also changes with the passage of time. Applying intersequence analysis method to financial risk prediction can greatly improve efficiency and save cost and has a wide application prospect.

## 2. Materials and Methods

### 2.1. Relevant Theories Based on Risk Prediction Model Design

Risk assessment in a broad sense is equivalent to risk management, including target determination, risk identification, risk assessment (risk valuation, risk analysis, and risk evaluation), and risk response. Risk assessment can be directly divided into risk valuation, risk analysis, and risk evaluation. Risk assessment in a narrow sense is a process of measuring, analyzing, judging, and ranking risks on the basis of risk identification, including risk valuation, risk analysis, risk evaluation, and other steps. It is the main basis for risk response and risk control. Due to the accuracy and applicability of different types of combined forecasting models, researchers have carried out many effective practical design and exploration studies and have also achieved many effective results in theoretical methods and practical applications [13].  Figure 1 shows the flowchart of the occurrence of international trade risks.

However, due to the universality of time series data encountered in actual production and life, as well as the complexity and variability of time series data itself, it is still very difficult to find a model that is suitable for all time series data and has good prediction ability.

#### 2.1.1. Basic Theory of Random Time Series

Time series refers to a series of ordered data formed by arranging and recording certain statistical indicators in chronological order [14]. Time series analysis is to analyze and study the abovementioned time series, study a model that can describe the change and development law of this phenomenon, and use the established model to predict its future development trend.

In statistics, the time series of a random event is usually a group of random variables arranged in chronological order:

(1) $$\begin{array}{c} X_{1},X_{2},\ldots ,X_{t}. \end{array}$$

To describe, abbreviated as {*X*_*t*_, *t* ∈ *T*}, *T* is a collection on the timeline. When there are *n* ordered detection values, use

(2) $$\begin{array}{c} x_{1},x_{2},\ldots ,x_{n}. \end{array}$$

In this way, the detection value sequence with the sequence length of *n* in the above formula is represented.

Stock price, gross national product, unemployment rate, and other data change with time and have time order. A series of variables arranged in time order are called time series [15]. Time series are data sets recorded at fixed time intervals. Time series has many aspects at the same time. The order of time series data is not easy to change. There is no regularity in the time series. If the random characteristics of a random process do not change with time, we call the process stationary. If the random characteristics of the random process change with time, the process is said to be nonstationary. The order of time series data cannot be easily changed. For those observations that are related to each other between the front and rear data, the order of their arrangement should be strictly observed, because there are usually regularities between the front and rear variables, so the time series data does not. It is suitable for analysis by ordinary statistical methods.

Based on the previous research, this paper found that when studying time series, the more stable the series is, the better the results will be [16]. Let a time series be {*X*_*t*_,  *t* ∈ *T*}, take *t*, *s* ∈ *T* arbitrarily, *T* is the set of time, so the expression by the autocovariance function is

(3) $$\begin{array}{c} \gamma \left(t,s\right)=E\left(X_{t}-\mu_{t}\right)\left(X_{s}-\mu_{t}\right). \end{array}$$

The autocovariance function parameter of time series {*X*_*t*_} is *ρ*(*t*, *s*), and its expression is

(4) $$\begin{array}{c} \rho \left(t,s\right)=\frac{\gamma \left(t,s\right)}{\sqrt{{\text{DX}}_{t}\cdot {\text{DX}}_{s}}}=\frac{\gamma \left(t,s\right)}{\sqrt{E{\left(X_{t}-\mu_{t}\right)}^{2}\cdot E{\left(X_{s}-\mu_{s}\right)}^{2}}}, \end{array}$$

where *μ*_*t*_ is the mean function of sequence {*X*_*t*_} at time *t*. Therefore, the above series become strictly stable time series. Only when the statistical characteristics of the series do not change with time can we achieve a stable time series.

Let a time series be {*X*_*t*_}, take any ∀*t*_1_, *t*_2_,…, *t*_*m*_ ∈ *T*, *T* is the set of time, and for any integer *m*, *τ*, we have

(5) $$\begin{array}{c} F_{t_{1},t_{2},\ldots ,t_{m}}\left(x_{1},x_{2},\ldots ,x_{m}\right)=F_{t_{1}+\tau ,t_{2}+\tau ,\ldots ,t_{m}+\tau }\left(x_{1},x_{2},\ldots ,x_{m}\right). \end{array}$$

While satisfying the above conditions, the strictly stable time series of time series {*X*_*t*_} is obtained.

#### 2.1.2. Fundamentals of Neural Networks

This paper will take BP neural network as an example to introduce this part. In recent years, great progress has been made in theoretical research based on artificial neural network, which is mainly used in many aspects such as function approximation, pattern recognition, classification, and data compression [17]. In artificial neural network, due to the research on the correction method of multilayer network connection weight, this is a new training method of multilayer feedforward neural network. The network model using this algorithm for error correction is called BP neural network model.  Figure 2 shows the basic model of BP neural network.

The learning of BP neural network algorithm consists of two processes: one is the forward output of signal and the other is the reverse output of error. In the process of forward output, the sample data is transmitted to the input layer, processed by each hidden layer in the middle, and then transmitted from the output layer [18]. If the output from the output layer is inconsistent with the desired output, enter the output process in the direction of error. The reverse output of the error is to transmit the error output from the output layer to the hidden layer in some form and finally to the input layer by layer. The error signal is used as the basis for modifying the weights of each unit, and the two processes and the adjustment process of the weights of each layer are carried out over and over again until the output error of the neural network is reduced to the set value or reaches a preset number of times.

Let *x*_1_, *x*_2_,…, *x*_*n*_ represent *n* input values, *ω*_1_, *ω*_2_,…, *ω*_*m*_ represent *m* weights, ∑*ω*_*i*_*x*_*i*_ represents the weighted sum of input signals of artificial neurons, *θ* represents the threshold, and *y* represents the output of neurons. When the value of ∑*ω*_*i*_*x*_*i*_ is greater than that of *θ*, the artificial neuron will be activated, and the output at this time is expressed as

(6) y=f∑ωix−iθ.

Among them, *f* the table shows the functional relationship between the output and input of artificial neurons. The transfer function selected by BP neural network is hyperbolic tangent function, expressed as

(7) $$\begin{array}{c} f\left(x\right)=\frac{e^{x}-e^{-x}}{e^{x}+e^{-x}}. \end{array}$$

BP neural network, as a multilayer feedforward neuron network with one-way propagation, generally consists of an input layer, an intermediate layer, and an output layer, and each layer is connected in sequence. Each layer consists of several artificial neurons, and all the neurons in each layer are completely connected, but there is no connection among the neurons in the same layer, and the output of the neurons in the previous layer is used as the input of the neurons in the next layer [19]. Therefore, when the input sample, the connection weight *ω*_*ij*_ between the input layer and the middle layer, and the threshold *θ*_*j*_ of each unit in the middle layer calculate the input *s*_*j*_ of each unit in the middle layer, then the transfer function can calculate the output *b*_*j*_. The following is the expression of the formula:

(8) $$\begin{array}{c} s_{j}=\sum_{i=1}^{n}\omega_{ij}a_{i}-\theta_{j},\\ b_{j}=f\left(s_{j}\right),\;j=1,2,\ldots ,p. \end{array}$$

After the connection weight is calculated, the input *l*_*t*_ between each unit can be calculated, and then the actual output value *c*_*t*_ can be calculated through the transfer function. The following is the expression of the formula:

(9) $$\begin{array}{c} l_{t}=\sum_{j=1}^{p}\upsilon_{jt}b_{j}-\gamma_{t},\\ c_{t}=f\left(l_{t}\right),\;t=1,2,\ldots ,q. \end{array}$$

Then calculate the correction error *d*_*t*_^*k*^ as follows:

(10) $$\begin{array}{c} d_{t}^{k}=\left(y_{t}^{k}-c_{t}\right)\cdot c_{t}\left(1-c_{t}\right),\;t=1,2,\ldots ,p. \end{array}$$

After obtaining the above data, you can calculate the next new connection weight *υ*_*jt*_ and threshold *γ* between the middle layer and the output layer:

(11) $$\begin{array}{c} \upsilon_{jt}\left(N+1\right)=\upsilon_{jt}\left(N\right)+\alpha \cdot d_{t}^{k}\cdot b_{j},\\ \gamma_{t}\left(N+1\right)=\gamma_{t}\left(N\right)+\alpha \cdot d_{t}^{k}. \end{array}$$

In the above formula, 0 < *α* < 1 is the learning coefficient of the BP neural network, and *N* is the number of times of network learning.

#### 2.1.3. Relevant Theories of International Trade Risk

International trade risk refers to the relevant possibility that international objects suffer losses due to various unforeseen factors in the process of international trade [20]. Moreover, this possibility exists objectively in a certain environment, and whether it can be turned into a fact has great uncertainty [21].  Figure 3 shows the evaluation interval chart of enterprises' international trade risk indicators.

The final output of risk management is alarm information and relevant countermeasures and suggestions. This prediction information is the useful information of the original information after inference and processing. It is a kind of information with high density and warning. To manage foreign trade risks of enterprises, we must master information, process information, and transform information. Therefore, we must choose the principle of information theory, grasp the law of information movement, eliminate untrue information and useless information, and transform the original information into conscious information and useful information for decision-making. Feedback control is widely used in enterprise foreign trade risk management. For example, once the product demand in the international market changes, the enterprise continuously adjusts its product structure and marketing strategy according to the changed market demand. The enterprise should strive for the initiative in the international market competition. Therefore, it is necessary to combine feedback control and feedforward control to conduct compound control of international market risks, so as to seize opportunities in time and resolve foreign trade risks as soon as possible [22]. Decision time is the time needed for decision makers to make correct decisions based on decision information. The implementation time is the time required to turn the decision into action and implement it. The effect time is the time required to produce the effect after the implementation of the decision. There are many factors causing the emergence of national risks, but many risk factors are directly related to history. It is necessary to pay more attention to international macrofactors in order to analyze the factors causing national risks [23].

### 2.2. Time Series Analysis of Risk Prediction

The risk limit is generally expressed by four numerical values, which are called check values. Taking these four check values as the limit, it means that the international trade operation state of the enterprise is in “dangerous state,” “semidangerous state,” “seminormal state,” and “normal state” [24]. For risk prediction, we need to know several time series to have a good grasp. First, information collection: the task of this stage is to collect relevant information according to specific prediction phenomena. The focus is on the scope of information collection, and the coverage should be as wide as possible, including various factors affecting the international trade of enterprises. Then, information screening: at this stage, multiple analytical studies are performed on all the information collected. Second, the evaluation of information: once the screening and filtering work is completed, further evaluation must be carried out to determine the actual importance of these information items. Then, the setting of the critical value, together with relevant experts, determines the critical value of the predictive index according to experience and theory. If some parameters of information approach reach this critical value, it means that there will be international trade risk events. Finally, report risk: once a specific parameter approaches or reaches a critical value, the system will report an upcoming event at an appropriate time.

When establishing the international trade risk management model, it should be considered that there should be submodels to deal with these two kinds of information in the model. As the enterprise international trade risk management system is often a very complex system, the information to be collected and processed includes all kinds of quantitative and qualitative information.

The formulation of risk measurement scheme should exist in the whole process of international trade risk measurement. This is because, in innovative international trade projects, many transactions are unknown. The only way to grasp this uncertainty is to constantly redefine the project and embed this redefinition deeply into the project infrastructure. The development of risk measurement scheme can naturally control the supervision of the project. Of course, the key to the risk measurement scheme is before the trade project, and the current risk measurement is the most important. According to the scheme design, the measurement process is fully invested in the trade project, which makes the control of international trade risk more effective.

Therefore, in the test process, the most important thing is to collect and process all kinds of information related to this phenomenon in the system. The quality of this work is directly related to the correctness of the conclusion.

### 2.3. Establishment and Analysis of the Risk Prediction Model

International trade risk mainly refers to the risk occurring in the business process of international trade. For example, in the preparation process before the transaction, the credit risk was caused by the distortion of market research. This is because international trade is an activity closely dependent on the environment, especially on the international environment. Therefore, there are many risk factors inducing international trade. The fierce competition in the international market and the complex and changeable international and domestic environment make the risk factors of international trade more complex and difficult to grasp accurately. As a result, international trade risk events often occur and lead to significant risk losses. For the establishment of the model, this paper designs it from both quantitative and qualitative aspects, so as to better realize the organic prediction and dynamic analysis of international trade risk. After comprehensively analyzing various index data and parameters, the interference items and errors are screened and filtered, which greatly improves the accuracy of the risk prediction model and reflects the reliability and practicability of the model [25].  Figure 4 shows the basic risk management model.

The first aspect: weighted improvement, which can make full use of the latest useful information and reduce randomness. The second aspect: add an interference factor. The purpose of the two improvements is to improve the accuracy of foreign trade risk prediction on the one hand and to reflect the decision-maker's participation in risk prediction by adding interference factors on the other hand. To deal with qualitative factors, a multiparty comprehensive survey method can be used, which can make probability estimates for a large number of nontechnical factors that cannot be quantitatively analyzed and inform experts of the results of probability estimates, giving full play to the role of information feedback and information control, so that scattered experts opinions gradually converge on a coordinated evaluation result.

The main basis of prediction is information, so a sensitive prediction information system must be established. Prediction information is the result of the transformation from original information to symptom information. The original information includes historical information and instant information, as well as actual information, judgment information, domestic information, international information and international trade, and economic and social information related to enterprises. Theoretically, if a sequence of observations contains nonstationary deterministic information, it can be extracted simply, effectively, and fully as long as it has been subjected to multiple differential operations. However, the more the number of differential operations, the better. Excessive differential operations will lead to the loss of useful information. Therefore, in the actual calculation, the differential operation of appropriate order should be selected to avoid over differential. In this paper, the ARIMA model is used to study the error of time series. The time series {*x*_*t*_} is as follows:

(12) $$\begin{array}{c} x_{t}=\beta_{0}+\beta_{1}t+\varepsilon_{1}. \end{array}$$

Make a difference on the sequence, and observe the stationarity and variance of the sequence after the difference. First, the first-order difference is as follows:

(13) $$\begin{array}{c} \nabla x_{t}=\beta_{1}+\varepsilon_{t}-\varepsilon_{t-1}. \end{array}$$

The differenced series is stationary, and its variance form is expressed as

(14) $$\begin{array}{c} \text{Var}\left(\nabla x_{t}\right)=\text{Var}\left(\varepsilon_{t}-\varepsilon_{t-1}\right)=2\sigma_{\varepsilon }^{2}. \end{array}$$

Then calculate the second-order difference:

(15) $$\begin{array}{c} \nabla^{2}x_{t}=\varepsilon_{t}-2\varepsilon_{t-1}+\varepsilon_{t-2}. \end{array}$$

After calculation, it is found that the second-order difference is also stable, and its variance form is

(16) $$\begin{array}{c} \text{Var}\left(\nabla^{2}x_{t}\right)=\text{Var}\left(\varepsilon_{t}-2\varepsilon_{t-1}+\varepsilon_{t-2}\right)=6\sigma_{\varepsilon }^{2}. \end{array}$$

Since the second-order difference is three times that of the first-order difference, which will reduce the accuracy of the prediction model, in general, this paper chooses to use the inverse autocorrelation function of the sequence to judge the excessive difference of the sequence.  Figure 5 shows the model modeling framework of ARIMA.

## 3. Result Analysis and Discussion

With the liberalization of the right to operate import and export, domestic enterprises have no restrictions on the right to operate import and export. As long as there is demand, they can conduct import and export transactions by themselves. The demand of Shanghai enterprises as import and export agents in the traditional sense is decreasing. The business of the enterprise is gradually changing from acting as import and export agent in the initial period to self-supporting import and export. It is breaking the original situation, extending the service chain of the enterprise, expanding commodity sales channels, establishing its own import and export commodity sales network, consolidating the resource integration ability of logistics and capital flow in the import and export business process, and extending the diversification of import and export commodities at different levels. To this end, the following experiments are carried out to investigate the practical performance of the analytical model.  Figure 6 is a graph of profitability indicators for general companies.

From the graph, we can observe that the slope of the rate of return is slightly higher, which indicates that the business of enterprises has obvious seasonality. In fact, this phenomenon is not difficult to understand, because traditional festivals in China are concentrated in the first half of the year, especially the stimulation of consumption brought by the Spring Festival is unspeakable. Although the volatility of operating profit margin and net profit margin in different time dimensions becomes smaller, it also shows seasonal changes. This means that the profitability index is very suitable for forecasting with time series. On this basis, this paper has a basic basis for the prediction of the model.

Enterprise risk management is to analyze and evaluate the risks existing in the process of enterprise development and take corresponding measures to deal with the risk process to achieve a certain development. In the process of enterprise development, its internal risk refers to the change of interests caused by the limitation of its own operating ability or the constant change of its operating environment during the long-term development of an enterprise, which may lead to the failure of related activities in the process of operation of an enterprise. The purpose of risk management is to help managers choose a suitable goal. The selection of goal is based on the intention of the enterprise, and the size of Guangsheng's risk is also adaptive.  Figure 7 shows the performance of model risk prediction under Shanghai Stock Index.

In the empirical analysis based on the Shanghai Composite Index data in each time dimension, the line chart not only shows the data fitting situation of the combined forecasting model in the training process, but also shows the actual forecasting effect of the combined forecasting model on the test data set. The combined prediction model shows the best model effect, which is reflected in its lowest error index value. The model effect of the uncertain combination prediction model based on fuzzy theory is better than the compared model, which reflects that the uncertain combination prediction model based on time series theory constructed in this paper is a feasible modification to the time series model.

The purpose of risk management is to help managers choose a suitable target. The target selection is based on the intention of enterprises, and the risk of Guangsheng is also adaptive. Stabilize the original sequence. If a nonstationary time series is used to build a model, it is easy to have a false regression problem; that is, even if there is no relationship between the original input sequence and the fitted sequence, there is a significant correlation between them. To establish a regression model, when building a time series model, it is necessary to make the time series stationary. Compared with the time series models and theories in traditional statistics, the main difference between the fuzzy time series models is the processing logic of language variables.

Time series analysis provides a set of dynamic data processing methods with scientific basis. This method is mainly described by using corresponding mathematical models for various types of data. Then through the analysis and research of the model, we can understand the internal structure and complex characteristics of the data in essence. Prediction is to infer and measure the future development and changes of things. Economic prediction is based on a certain time series. In order to achieve the prediction accuracy and the best possible fitting accuracy, however, it is difficult to obtain satisfactory prediction results by using a single prediction method. In order to make full use of the advantages of various models and achieve the optimal prediction results, various single prediction methods can be organically combined. The combined forecasting model based on time series model and its application are discussed.

## 4. Conclusions

The model proposed in this paper optimizes the structure of the design model with the support of ARIMA algorithm and BP neural network algorithm and has good accuracy and error control for different time series. Due to the different characteristics of various prediction methods, the prediction effect also changes with the passage of time. Applying intersequence analysis method to financial risk prediction can greatly improve efficiency and save cost and has a wide application prospect. The model optimizes the structure of the design model with the support of ARIMA algorithm and BP neural network algorithm, and has good accuracy and error control for different time series. The purpose of establishing the time series prediction model is to improve the prediction accuracy of the model, and it is also an effective way to enhance the practicability of the prediction model. Applying intersequence analysis method to financial risk prediction can greatly improve efficiency and save cost and has broad application prospects. However, the research still has some limitations. Due to the different characteristics of various prediction methods, the prediction effect will also change with the passage of time.

## Figures and Tables

**Figure 1:** Flowchart of the occurrence of international trade risks.

**Figure 2:** Basic model of BP neural network.

**Figure 3:** Evaluation interval chart of international trade risk indicators.

**Figure 4:** Basic model diagram of risk management.

**Figure 5:** ARIMA model modeling architecture diagram.

**Figure 6:** The profitability index of general enterprises.

**Figure 7:** Model risk prediction performance chart under the Shanghai Composite Index.

## Data Availability

The data used to support the findings of this study are available from the corresponding author upon request.
